# Propofol inhibits migration and induces apoptosis of pancreatic cancer PANC-1 cells through miR-34a-mediated E-cadherin and LOC285194 signals

This article has been retracted.

**DOI:** 10.1080/21655979.2020.1754038

**Published:** 2020-04-17

**Authors:** Hongwei Wang, Hongmei Jiao, Ziru Jiang, Renyi Chen

**Affiliations:** a Department of Anesthesia, Linyi Cancer Hospital, Linyi, Shandong, China; b External Abdominal Section, Linyi Cancer Hospital, Linyi, Shandong, China

**Keywords:** Pancreatic cancer, microRNA-34a, long non-coding RNA LOC285194, E-cadherin, apoptosis, migration

## Abstract

Propofol has exhibited potent antitumor activity in pancreatic cancer cells *in vitro* and *in vivo*. The study aimed to investigate the anti-tumor mechanisms of propofol on pancreatic cancer PANC-1 cells *in vitro*. PANC-1 cells were exposure to concentration 20 μg/ml of propofol for 72 h. Long non-coding RNA LOC285194 siRNA LOC285194 siRNA, E-cadherin siRNA and microRNA-34a (miR-34a) inhibitor were used to investigate the effect of propofol on PANC-1 cells. miR-34a and LOC285194 were analyzed by quantitative real-time PCR (qRT-PCR). Pro-apoptotic protein bax, cleaved-caspase-3 and anti-apoptotic protein bcl-2 were analyzed by Western blot. Cell viability and cell apoptosis were detected by MTT and TUNEL staining, respectively. Cell migration was detected by wound-healing assay. The results showed that propofol upregulated miR-34a expression, which, in turn, upregulated LOC285194 expression, resulting in PANC-1 cell apoptosis and growth inhibition. In addition, propofol upregulated miR-34a expression, which, in turn, upregulated E-cadherin expression, resulting in cell migration inhibition. Our research confirmed that propofol-induced cell apoptosis and inhibited cell migration in PANC-1 cells *in vitro* via promoting miR-34a-dependent LOC285194 and E-cadherin upregulation, respectively.

## Introduction

Pancreatic cancer is the most fatal malignancies among all digestive system tumors, and it will be the second most frequent cause of cancer-related deaths within the next 10 years [1]. Although surgery remains the best choice for pancreatic cancer treatment, more than 80% of patients present with an unresectable primary tumor and distant metastasis at the time of diagnosis, a point in which surgical or chemotherapeutic interventions have minimal benefit [2]. Despite improvements in surgical techniques and adjuvant medical therapy, the 5-year survival rate is less than 5% [3]. Therefore, understanding the metastatic mechanisms can lead to better prevention and treatment of pancreatic cancer. Alteration of epigenetic pathways and changes in the tumor microenvironment is an emerging mechanism to initiate pancreatic cancer metastasis [4]. In addition, the shedding pancreatic cancer cells, also known as circulating tumor cells (CTCs), from the primary focus can enter into the bloodstream and transport to other parts of the body to seed new tumors [5]. Pancreaticoduodenectomy can result in the risk of squeezing and shedding of the cancer cells into the portal vein and subsequently cause a liver metastasis [6]. Therefore, inhibiting circulating tumor cells in the bloodstream could effectively inhibit metastasis and growth of pancreatic cancer cells.

Recent evidences indicated that anesthesia, such as local anesthetics or general anesthesia can inhibit cancer cell proliferation and reduce the risk of recurrence by kill tumor cells [7–11]. Propofol is one of the most popular intravenous anesthetic agents for induction and maintenance of anesthesia in China. It has recently been indicated that propofol shows obvious antitumor effect through different mechanisms. For example, propofol could inhibit *in vitro* cell growth and invasion by upregulating miR-140-5p in gastric cancer cells [12]. In human colon cancer cells *in vitro* and *in vivo*, propofol exerts its anti-tumor effect by activating WIF-1 and suppressing Wnt pathway [13]. In lung cancer A549 cells *in vitro*, propofol inhibited cell growth, migration and invasion by regulating miR-372/Wnt/β-catenin pathways [14]. In breast cancer MCF7 and MDA-MB-231 cells *in vitro*, propofol reduces cell migration and invasion by silencing NET1 expression [15]. A recent study reported that serum from patients receiving propofol anesthesia for colon cancer surgery inhibited proliferation and invasion of LoVo cells and induced apoptosis in vitro [16], suggesting that propofol might affect metastasis in patients with colon cancer. Recent studies have demonstrated that attenuate pancreatic cancer cells malignant potential via different mechanisms. Liu et al [17] reported that propofol effectively attenuates invasion of PANC-1 cells by miR-21/Slug pathway. Chen et al [18] reported that propofol suppressed migration of pancreatic cancer cells *in vitro* and i*n vivo* via targeting NMDA receptor. However, there is currently no clear mechanism to explain the roles of propofol in cancer cells. Thus, the identification of molecular targets provides theoretical basis for application of propofol in clinical anesthesia or antitumor therapy.

Accumulating evidence demonstrates that lncRNAs could play an important role in regulation of cell growth and apoptosis as well as cancer progression and metastasis. Long non-coding RNA LOC285194 (LOC285194) has shown a potential tumor-suppressor function in several types of human cancers, such as osteosarcoma [19], colorectal cancer [20] and non-small cell lung cancer [21]. Clinical data have demonstrated that, expression of LOC285194 in was significantly lower, and lower LOC285194 expression was closely correlated with clinical stage, lymphnode metastasis, liver metastasis and poor overall survival in patients with pancreatic cancer tissues [22]. Experimental research found that LOC285194 overexpression inhibited cell proliferation and induced apoptosis in vascular smooth muscle cells (VSMCs) *in vitro, and vice versa* [23]. In gastric cancer MKN45 and HGC-27 cells *in vitro* and *in vivo*, LOC285194 overexpression suppressed cell proliferation and promoted cell apoptosis [24].

Numerous studies have demonstrated that miRNAs play important roles in cancer development by regulating the expression of various oncogenes and tumor-suppressor genes [25]. Among the miRNAs, the miR-34a is a key regulator of tumor suppression, controlling cell cycle, differentiation and apoptosis, metastasis and chemoresistance [26]. In SW480 and HCT116 cells, miR-34a upregulated E-cadherin and the down-regulation of vimentin revealed the anti-EMT abilities of miR-34a [27]. miR-34 has been shown to regulate pancreatic cancer cell growth, invasion and metastasis *in vitro* and *in vivo* by targeting members of key signaling pathways [28–30]. Recent studies have demonstrated that propofol upregulated miR-34a expression and induced cell apoptosis in SH-SY5Y cells in vitro, and targeting miR-34 protected the SH-SY5Y cells from propofol-induced apoptosis [31,32].

In the present study, we aimed to investigate the effects of propofol on cell apoptosis and migration in pancreatic cancer PANC-1 cells and explored the mechanisms *in vitro*. We demonstrate for the first time that propofol-induced miR-34a dependent LOC285194 upregulation to induce PANC-1 cell apoptosis and inhibit cell viability. Propofol-induced miR-34a dependent E-cadherin upregulation to inhibit PANC-1 cell migration. Therefore, propofol might be against pancreatic cancer cells present in the bloodstream, by which inhibited pancreatic cancer cells growth and migration.

## Materials and methods

### Cell culture

The PANC-1 pancreatic cancer cell line was purchased from American Type Culture Collection (ATCC, Shanghai, China) and cultured as per the supplier’s instruction. The PANC-1 cells were cultured in Dulbecco’s modified Eagle’s medium (DMEM) supplemented with 10% fetal bovine serum (FBS) (Gibco, mexico), 5 U·mL−1 penicillin, 0.5 U·mL−1 streptomycin and 2 mm glutamine. in a 37°C incubator with a 5% CO_2_ humidified atmosphere.

### Transfection of miRNA inhibitor and small interfering RNA

MiR-34a inhibitors (anti-miR-34a), and a matched miRNA negative control (miR-NC) were synthesized and purified by Shanghai Genechem. (Shanghai, China). miR-NC, sense 5′-UUCUCCGAACGUGUCACGTT-3′, antisense 5′-ACGUGACACGUUCGGAGAATT-3′; and anti-miR-34a 5′-ACAACCAGCUAAGACACUGCCA-3′. Small interfering RNA-E-cadherin (E-cadherin siRNA), small interfering RNA-LOC285194 (LOC285194 siRNA), and negative control (NC) were purchased from Shanghai Jikai Gene Chemistry Co (Shanghai, China). Briefly, PANC-1 cells (2 × 10^4^ cells/mL) were seeded into 10-cm Petri dishes. Twenty-four hours later, siRNAs were mixed with Lipofectamine 3000 (Invitrogen, Carlsbad, CA, USA) at 1:2 ratio (siRNA: transfection reagent) in serum and antibiotic-free Opti-MEM medium (Life Technologies, Grand Island, NY). The transfection mix was incubated for 20 min at room temperature (RT) and then added to the cells. Cells were incubated at 37°C and collected 48-hr post-transfection to assess the LOC285194 and miR-34a by qRT-PCR and western blot for E-cadherin. The miR-34a inhibitor transfection was performed using the Invitrogen™ Lipofectamine® 3000 transfection reagent, according to the manufacturer’s instructions (Thermo Fisher Scientific Inc., Waltham, MA, USA). All the small RNAs and miR-34a mimic/inhibitor were used at a final concentration of 50 nM.

### Drug treatment

Propofol was purchased from Aldrich (Milwaukee, WI). Propofol was diluted in dimethyl sulfoxide (**DMSO**, Sigma, St. Louis, MO, USA) to a stock concentration of 1.78 mM, and stored in −20°C. PANC-1 cells were treated with concentration 20 μg/ml propofol for 72 h.

### RNA extraction and quantitative real-time PCR

The total RNA of PANC-1 cells was extracted according to the manufacture’s instructions provided in the Trizol kit (Invitrogen Inc., Shanghai, China). LOC285194 and miR-34a expression were detected using TaqMan microRNA assays (Life Technologies) in an Applied Biosystems 7500 Real-Time PCR System according to the manufacturer’s instructions. Experiments were performed in triplicate and U6 snRNA (U6) was used as an internal control to normalize LOC285194 or miR-34a. The relative expression levels were calculated using 2^−ΔΔCq^ method [33].

### Western blot

After the indicated treatment, the PANC-1 cells were washed and lysed and the proteins in the cell lysate were separated by centrifugation. The proteins were separated on 10% SDS-PAGE gel and then transferred to PVDF membranes (Bio-Rad) and immunoblotted with the mouse anti-E-cadherin (Cell Signaling) and anti-GAPDH antibodies (Santa Cruz Biotechnology). At last, the proteins were visualized using ECL-plus detection system (Pierce).

### MTT assay

PANC-1 cells were seeded into 96-well plates (5 × 10^3^ cells/well) for 24 h. Then, concentrations 20 μg/ml of propofol was added to the wells for 72 h. To detect the effect of LOC285194 or miR-34a or E-cadherin on propofol-induced cell growth and apoptosis in PANC-1 cells, the PANC-1 cells were transfected with LOC285194 siRNA or miR-34a inhibitor or E-cadherin siRNA or its controls for 24 h, then treated with concentrations 20 μg/ml of propofol. After 72 h, 20 µL of MTT (5 mg/mL, Sigma) was added into each well and incubated for another 4 h at 37°C. Absorbance was measured at 580 nm with a SpectraMax Plus MicroPlate Reader (Molecular Devices, Sunnyvale, CA).

### TUNEL staining

To detect apoptotic cells, the DeadEnd™ Colorimetric Apoptosis Detection System from Promega (Madison, WI) was used. The PANC-1 cells were transfected with LOC285194 siRNA or miR-34a inhibitor or E-cadherin siRNA or its controls for 24 h. Then, the cells were plated at a density of 1 × 10^6^ cells/well in 6-well plates and treated with 20 μg/ml of propofol for 72 h. Cell apoptosis was detected as the manufacture’s instruction. The total number of cells was counted using DAPI staining, and the average ratio of TUNEL-positive cells was calculated.

### Wound healing assay

The assay was performed using the Cytoselect wound healing kit (Cell Biolabs) according to the manufacturer’s instructions. The PANC-1 cells were transfected with LOC285194 siRNA or miR-34a inhibitor or E-cadherin siRNA or its controls for 8 h, then treated with concentrations 20 μg/ml of propofol for 24 h. After which the cells were inoculated at 1 x 10^4^/well in 6-well plates and cultured to confluence. Confluent cell monolayer was then scraped with a straight line using a 200 μl pipette. Five viewpoints were photographed at 0 h and 24 h after the scar was made. The mean migration distance was determined and analyzed using Image ProPlus version 6.0 software.

### Statistical analysis

Each experiment was repeated at least three times. Data were presented as means±standard deviation. Data were analyzed for statistical significance using the Student’s t-test using SPSS 22.0 soft (SPSS, USA). *P* < 0.05 was considered statistically significant.

## Results

### *Propofol-induced cell apoptosis* in vitro

Propofol is a widely used intravenous anesthetic shown to exert an anti-tumor effect by inducing cell apoptosis [14–17]. In this study, cell viability was markedly reduced by 20 μg/ml propofol exposure for 72 h compared with the untreated PANC-1 cells (Figure 1 A, *P* < 0.01). Percentage of apoptotic cells in the propofol-treated group was notably higher (*P* < 0.01, Figure 1(b)). Western blot results in Figure 1(c) showed that expression of pro-apoptotic cleaved caspase-3 and Bax was up-regulated after propofol exposure, whereas expression of anti-apoptotic Bcl-2 was down-regulated after propofol exposure.

**Figure 1.** **Propofol-induced LOC285194-dependent PANC-1 cell apoptosis**. PANC-1 cells were transfected with LOC285194 siRNA or NC siRNA with/without propofol (20 μg/ml) treatments for 72 h. a, Cell viability by CCK-8. b, Percentage of apoptotic cells by flow cytometry assay. c, Expression of apoptosis-related proteins by Western blot analysis. vs untreated, ^a^p<0.01, vs propofol or propofol+NC siRNA, ^b^p<0.01, vs untreated, ^c^p> 0.05.

### Propofol-induced cell apoptosis through LOC285194 upregulation

The LOC285194 siRNA or NC siRNA transfected PANC-1 cells were exposed to 20 μg/ml propofol for 72 h, and then cell viability and apoptosis were analyzed. Results showed that effects of propofol exposure on PANC-1 cells could be significantly reversed by LOC285194 siRNA transfection to target LOC285194, as evidenced by decreased cell viability (*P* < 0.01, Fig. 1.A), increased apoptotic cells (*P* < 0.01, Fig. 1.B), down-regulation of cleaved caspase-3 and Bax, and up-regulation of Bcl-2 (*P* < 0.01, Fig. 1.C)

### Propofol-induced cell apoptosis through upregulating miR-34a -dependent LOC285194 expression

MiR-34a acts as a tumor suppressor in several cancers, including pancreatic cancer, by controlling the expression of target proteins involved in cell cycle, differentiation and apoptosis [34,35]. We next investigated whether propofol-induced LOC285194-dependent miR-34a upregulation. To test its involvement in LOC285194 induction, we first evaluated miR-34a activation during propofol treatment of PANC-1 cells by qRT-PCR assay. PANC-1 cells were exposed to 20 μg/ml propofol for 72 h, both expression of miR-34a and LOC285194 was significantly increased compared with the untreated PANC-1 cells (*P* < 0.01, Figure 2(a)). We further examined whether the up-regulation of LOC285194 depends on miR-34a. The PANC-1 cells were transfected with miR-34a inhibitor to block miR-34a expression, then exposure to 20 μg/ml propofol for 48 h. Propofol-induced LOC285194 upregulation was almost completely blocked following miR-34a downregulation in the PANC-1 cells (*P* < 0.01, Figure 2(a)).

**Figure 2.** Propofol-induced cell apoptosis by miR-34a-dependent LOC285194 induction. PANC-1 cells were transfected with miR-34a inhibitor or NC inhibitor with/without propofol (20 μg/ml) treatments for 72 h. a, Expression of miR-34a and LOC285194 was detected by qRT-PCR assay. b, Cell viability by CCK-8. c, Percentage of apoptotic cells by flow cytometry assay. d, Expression of apoptosis-related proteins by Western blot analysis. vs untreated, ^a^p<0.01, vs propofol, ^b^p<0.01, vs untreated, ^c^p> 0.05.

To reveal the functional role of **m**iR-34a in propofol-induced cell viability and cell apoptosis, the miR-34a inhibitor or NC transfected PANC-1 cells were exposed to 20 μg/ml propofol for 72 h, and then cell viability and cell apoptosis were analyzed. The results showed that miR-34a inhibitor-transfected cells restored propofol-induced cell viability (*P* < 0.01, Figure 2(b)) and reduced propofol-induced cell apoptosis (*P* < 0.01, Figure 2(c)) compared with the NC inhibitor transfected PANC-1 cells. However, restoration of LOC285194 expression by Lv-LOC285194 transfection increased miR-34a inhibitor/propofol treated PANC-1 cells (data not shown). miR-34a inhibitor alone failed to affect cell apoptosis and viability. Also, as shown in Figure 2(d), miR-34a inhibitor transfection significantly suppressed caspase-3 processing/activation and Bax expression, and upregulation of Bcl-2 expression.

### Propofol inhibits cell migration through upregulating E-cadherin

E-cadherin is one of the well-studied founding members of the superfamily and a potent tumor suppressor because downregulation of E-cadherin is often found in malignant epithelial cancers [34]. Loss of E-cadherin in cancer cells leads to metastatic dissemination and activation of several EMT transcription factors [36]. As shown in Figure 3a, E-cadherin protein was low expressed in the PANC-1 cells, and significantly increased in PANC-1 cells exposure to 20 μg/ml propofol for 72 h by western blot assay. Furthermore, propofol treatment exhibited reduced motility as determined by wound healing assays (Figure 3(b)). To determine whether E-cadherin upregulation impaired cell motility in PANC-1 cells following propofol treatment, E-cadherin siRNA was used to targeting E-cadherin expression in the PANC-1 cells. As shown in Figure 3(a), transient expression of E-cadherin siRNA blocked propofol-induced E-cadherin expression in the PANC-1 cells, and resulted in a significant reduction in cell motility ability compared with that observed in NC siRNA control group in PANC-1 cells by wound healing assays (Figure 3(b)). Although propofol treatment induced LOC285194 upregulation, however, targeting LOC285194 failed to influence propofol-induced PANC-1 cell migration and invasion (Figure 3(b)), suggestive of a specific role of E-cadherin signal in regulating migration.

**Figure 3.** Propofol inhibits cell migration by inducing E-cadherin. PANC-1 cells were transient expression of E-cadherin siRNA or LOC285194 siRNA or its control, then exposure to 20 μg/ml propofol for 72 h. a, E-cadherin protein expression was detected by Western blot assay. b, Cell migration was detected by wound healing assays. vs untreated (24 h), ^a^p<0.01, vs propofol (24 h), ^b^p<0.01, vs propofol (24 h), ^c^p> 0.05.

### Propofol inhibits cell migration by upregulating miR-34a -dependent E-cadherin expression

miR-34a is involved in certain EMT-associated signal pathways to repress tumorigenesis, cancer progression, and metastasis [34]. We next examined whether the up-regulation of E-cadherin depends on miR-34a. The PANC-1 cells were transfected with miR-34a inhibitor to block miR-34a expression, then exposure to 20 μg/ml propofol for 72 h. The results showed propofol-induced E-cadherin upregulation was completely blocked following miR-34a downregulation in the PANC-1 cells (Figure 4(a)).

**Figure 4.** Propofol inhibits cell migration by miR-34a-dependent E-cadherin expression. PANC-1 cells were transfected with miR-34a inhibitor or NC inhibitor with/without propofol (20 μg/ml) treatments for 72 h. a, E-cadherin protein expression was detected by Western blot assay. b, Cell migration was detected by wound healing assays. vs untreated, ^a^p<0.01, vs propofol, ^b^p<0.01.

To reveal the functional role of **m**iR-34a in propofol-induced cell migration, the miR-34a inhibitor or NC transfected PANC-1 cells were exposed to 20 μg/ml propofol for 72 h, cell migration was detected by wound healing assays. The results showed that targeting miR-34a expression with miR-34a inhibitor resulted in significantly increased cell migration compared with that observed in NC inhibitor transfected PANC-1 cells. Also, as shown in Figure 4(b), miR-34a inhibitor transfection significantly blocked propofol-induced E-cadherin upregulation compared with that observed in NC inhibitor transfected PANC-1 cells. Although propofol treatment induced E-cadherin upregulation, however, targeting E-cadherin failed to influence propofol-induced PANC-1 cell viability and apoptosis (data not shown) suggestive of a specific role of **LOC285194** signal in regulating cell survival.

## Discussion

Apart from its anesthetic effects, propofol also exerts a number of non-anesthetic effects, such as reduction of oxidative damage [37], decreases pro-inflammatory cytokines [38], inhibits COX-2 and PGE_2_ functions and decrease surgery-induced neuroendocrine responses and cause less immunosuppression and recurrence of certain types of cancer [39,40]. *In vitro* and *in vivo*, propofol could inhibit invasion, migration, metastasis and induced apoptosis and cell cycle arrest of numerous cancer cells [12–18].

The studies in animals [41] and humans [42] indicated that the measured/predicted brain concentration of propofol during maintenance of surgical anesthesia is above 4 µg/ml, and as high as 20 µg/ml [43,44]. Thus, in the *in vitro* experiments, the doses of propofol used that are within the range of concentrations found in the human brain during surgical anesthesia are referred to as anesthetic doses.

In the present study, we used clinically relevant dose of propofol (concentration 20 μg/ml) for further study. PANC-1 cells treated with 20 μg/ml propofol for 72 h exhibited decreased cell viability and increased cell apoptosis in the PANC-1 cells *in vitro.*

It is known that caspase family and Bcl-2 family are the major families involved in apoptosis. Caspase-3 is the critical executioner to participating in ‘extrinsic’ and “intrinsic apoptosis process [45]. Bcl-2 or Bax is the key antiapoptotic or proapoptotic protein and is induced by stress stimulation [46]. In this study, we compared the expression of caspase-3, bax and Bcl-2 in propofol-treated PANC-1 cells and the untreated PANC-1 cells. The results support the observation that propofol-induced cell apoptosis as the levels of proapoptotic proteins caspase-3 and bax are significantly higher, and bcl-2 is significantly lower than the untreated cells.

LOC285194 has shown a potential tumor-suppressor function in several types of human cancers [19–21]. Furthermore, the tumor suppression function of loc285194 was also suggested by knockdown experiments, which showed an increased cell proliferation and decreased cell apoptosis [47]. In this study, expression of LOC285194 was upregulated in the PANC-1 cells exposure to propofol treatment. However, after LOC285194 was blocked in PANC-1 cells, the propofol-induced cell apoptosis was significantly decreased and the cell viability was increased. The results support the observation that LOC285194 downexpressing inhibited propofol-induced upregulation of caspase-3 and bax, and reversed propofol-induced downregulation of bcl-2. These data indicated that propofol inhibited cell viability and promoted cell apoptosis via upregulating LOC285194 expression in the PANC-1 cells.

Propofol has reported to inhibit cell proliferation and migration of PANC-1 cells in vitro by downregulation of integrin β1, ERK1/2, MMP2 and MMP9 [48]. However, in oral squamous cell carcinoma (OSCC) cells, propofol treatment significantly promoted cell migration and invasion by up-regulation of Snail and down-regulation of E-cadherin [49]. It is suggested that what the propofol functions may be related to different tissues and cell specificities. In this study, propofol treatment significantly inhibits PANC-1 cell migration *in vitro*, followed by the upregulation of E-cadherin expression. However, cell migrative ability was reversed in the E-cadherin downexpressing PANC-1 cells following by propofol exposure. In addition, LOC285194 downexpression failed to affect propofol-induced cell migration in the PANC-1 cells, and E-cadherin downexpression failed to affect propofol-induced cell viability and apoptosis in the PANC-1 cells. We, therefore, concluded that propofol inhibited cell migration by E-cadherin-dependent pathway. It is suggested that propofol might be suitable for anesthesia management in pancreatic cancer patients. Related clinical treatments have also confirmed that propofol anesthesia helps reduce postoperative complications and improve long-term survival of patients with pancreatic cancer [50–52].

Specifically, the following findings from cell culture models showed that miR-15a-5p [53], MicroRNA-582-5p [54] and miR-34a [55] were involved in propofol-induced neuron and astrocyte death, respectively; miR-21 was involved in propofol-induced inhibition of proliferation and epithelial–mesenchymal transition in breast cancer cells [56]; miR-495 was involved in propofol-induced inhibition of proliferation and metastasis in JEG-3 choriocarcinoma cells [57]. In this study, propofol treatment decreased cell migration followed by miR-34a and E-cadherin upregulation in the PANC-1 cells. However, when miR-34a was blocked by miR-34a inhibitor, propofol-induced cell apoptosis was decreased and migrative cells were increased. Furthermore, propofol-induced upregulation of LOC285194 and E-cadherin expression was inhibited. These data indicated that propofol promoted cell apoptosis by miR-34a-dependent LOC285194 upregulation, and propofol inhibited cell migration by miR-34a-dependent E-cadherin upregulation.

The disseminated tumor cells (DTCs) and circulating tumor cells (CTCs) have been detected in the peripheral blood of many cancer types, including colorectal cancer [58], breast cancer [59], hepatocellular cancer [60] and pancreatic cancer [61–63]. The DTCs and CTCs in the blood could be awakened after surgery, initiating metastasis [64]. According to our study above, propofol might kill the DTCs and CTCs in the bloodstream of the pancreatic cancer patients, which would play an important role to inhibit tumor cell growth and metastasis. In the future, we will investigate whether propofol could kill the DTCs and CTCs cells in the bloodstream of the pancreatic cancer patients. In addition, the effect and mechanisms of propofol on pancreatic cancer cells in vivo will also investigated.

## Conclusion

Our research confirmed that propofol induces cell death via miR-34a-mediated LOC285194 upregulation; Propofol inhibited PANC-1 cell migration via miR-34a-mediated E-cadherin upregulation. These data indicated that propofol might kill the pancreatic cancer cells in the bloodstream and serve as a therapeutic role for pancreatic cancer in the future.

## Highlight

1. Propofol promotes cell apoptosis and inhibits viability via upregulation of LOC285194 in PANC-1 cells
2. Propofol inhibits cell migration via upregulation of E-cadherin in PANC-1 cells
3. Propofol upregulates miR-34a-dependent LOC285194 and E-cadherin expression in PANC-1 cells
